The article "Kinetics and Isotherm Studies for Adsorption of Gentian Violet Dye from Aqueous Solutions Using Synthesized Hydroxyapatite" was published in 2023. Journal: J Environ Public Health.

# Kinetics and Isotherm Studies for Adsorption of Gentian Violet Dye from Aqueous Solutions Using Synthesized Hydroxyapatite

**DOI:** 10.1155/2023/7418770

**Published:** 2023-05-29

**Authors:** Dalia A. Ali, Fatma A. Saad, Hoda A. Elsawy

**Affiliations:** Department of Chemical Engineering, The British University in Egypt, El Shorouk City 11837, Egypt

## Abstract

Water is the most important resource for life, but it has been greatly exhausted over the past century as a result of the human population and environmentally harmful activities. The excessive quantity of dyes exists in the wastewater produced from the textile industries which is the main reason for serious human health and environmental problems. There are many dye removal techniques, and the most promising one is the adsorption technique. The novelty of this research is using unmodified synthesized hydroxyapatite (HAp) as an adsorbent for the removal of gentian violet (GV) dye from aqueous solutions as there are no sufficient data in the literature about using it in the adsorption of GV dye from aqueous solutions. Unmodified HAp was synthesized by a combined precipitation microwave method. The prepared adsorbent was characterized by scanning electron microscopy (SEM), energy dispersive X-ray (EDX), X-ray diffraction (XRD), Fourier transform infrared (FTIR) spectroscopy, and zeta potential analyses. The kinetic study showed that the pseudo-second-order (PSO) model was the best fitted model with the experimental data. Analysis of adsorption isotherms using different models showed that this adsorption system was better described by the Halsey isotherm with a maximum adsorption capacity (*q*_max_)  of 1.035 mg/g. The effects of experimental factors such as initial solution pH, initial dye concentration, adsorbent dose, and contact time were studied during the investigation of GV dye removal efficiency. The experimental results indicated that the maximum adsorption efficiency (99.32%) of the GV dye using HAp adsorbent was achieved at the following conditions: contact time = 90 min, pH = 12, initial GV dye concentration = 3 mg/L, and adsorbent dose = 1 g/L. The adsorption mechanism of the GV dye using HAp might be explained by the electrostatic interaction between the negatively charged surface of the HAp and the positively charged group of the GV dye. Thermodynamics study was performed on the adsorption process of GV dye from aqueous solutions using the synthesized HAp which revealed that this process was endothermic and spontaneous due to positive values of Δ*H* and Δ*S* and negative values of Δ*G*.

## 1. Introduction

Water is a vital natural resource for the survival of all living things, food production, economic development, and general quality of life. Nowadays, contamination of water is one of the greatest global problems. Water has been contaminated by the release of radioactive elements, sediments, organic and inorganic compounds, and pesticides, and both natural and anthropogenic processes, such as mining, industrial waste, and domestic sewage, have depleted this natural and valuable resource [1]. Consequently, the quality of freshwater has been seriously affected, leading to the modification and replacement of all freshwater elements [2]. According to some studies, by 2025, water shortages would affect about half of the world's population. According to a study published in November 2009, water demand in some developed regions of the world will exceed by 50% by 2030 [3]. Therefore, treatment of wastewater is extremely necessary as water is an essential element for the survival of living beings [4]. Textile plants emit a variety of environmentally harmful dyes and chemicals. Significant amounts of wastewater are processed in the dyeing and finishing industries. Natural and inorganic compounds are used to make pigments and dyes [5]. Saturated and dissolved solids, biological oxidation demand (BOD), chemical oxygen demand (COD), chemicals containing trace metals such as chromium (Cr), arsenic (As), copper (Cu), and zinc (Zn), and colors are all pollutants in the textile industry that can damage the atmosphere and cause health impacts [6]. The industrial dyes are highly stable, lethal, and cancer-inducing, which causes harmful effects on the human health and the ecosystems. GV is a synthetic cationic dye also known as basic violet 3 which belongs to the group of triarylmethane. This dye is used extensively in the textile industry to dye cotton, wool, silk, and nylon, in the manufacture of printing inks, and also as the biological stain, a dermatological agent in veterinary medicine. GV dye causes skin damage and even cancer in humans and other animals. Various techniques have been applied for the removal of dyes including membrane separation, ion exchange, biological degradation using various microorganisms, electrocoagulation, and adsorption [5]. Membrane technology has a good ability to reduce high dye rejection [7]. The membrane separation process occurs due to the transfer of molecules via membranes based on differences in concentration (Δ*C*), temperature (Δ*T*), pressure (Δ*P*), and energy (Δ*E*) [7]. Although this process is efficient for the removal of dyes from wastewater, it has many disadvantages as it needs high operating pressure (70 bar) which leads to an increase in the operating cost and it is not applicable to large flow rates of wastewater [7]. Dyes can be efficiently removed from wastewater through an ion exchange method. This separation method depends mainly on making strong interactions between the charged dye molecules and the functional groups existing on the surface of the ion exchange resin [8]. The disadvantage of this method is that it is not suitable to be used in the case of high concentrated dye wastewater as the resin gets easily fouled by dye particles and other solids in the wastewater [9]. In addition, the ion exchange method is nonselective and it is highly sensitive to the pH of the solution [9]. Electrocoagulation treatment process is described as the generation of metal ions from anodes hydrolyzed into metal hydroxides and the generation of hydrogen (*H*_2_) bubbles that occur at the cathode which help the coagulated matters float. Although this method is simple in its operation and removes dyes efficiently from wastewater, it produces large amounts of sludge [10]. Biological treatment method is mainly used for the removal of dissolved organic matters included in the textile wastewater and this treatment method depends on the temperature range, the ratio between the organic compounds, microorganisms, and dye loads, and the concentration of oxygen. This treatment method has many disadvantages, including the production of high amounts of sludge which requires further treatment and high operating cost [11]. Among the above-mentioned methods, adsorption becomes more promising due to its high removal efficiency, high adsorption capacity, nontoxicity, and its ability to be used for the same adsorption process for several times [11]. Agricultural wastes such as potato peels and avocado seed powder have been recently used as adsorbents for different types of dyes, as represented in Table 1 [12–14], but they need several pretreatment processes including washing, drying, sieving, and grinding before using them as adsorbents [15].

The article "Kinetics and Isotherm Studies for Adsorption of Gentian Violet Dye from Aqueous Solutions Using Synthesized Hydroxyapatite" was published in 2023. Journal: J Environ Public Health.

Also, there are other materials such as modified HAp that have been recently used for the adsorption of different types of dyes as represented in Table 2 [16]. HAp is a calcium phosphate used in various fields including medicine and chemistry, and it is identified as a good adsorbent material for the environmental processes due to its specific structure conferring ionic exchange property and adsorption affinity towards many pollutants such as heavy metal ions, phenols, and dyes [13, 14]. According to several recent studies mentioned in Tables 1 and 2 and based on the value of maximum adsorption capacity (*q*_max_) in mg/g, it is obviously noted that HAp/hydrolyzed polyacrylamide 75 adsorbent with *q*_max_ = 435.6 mg/g is better than potato peels (*q*_max_ = 33.55 mg/g) and yellow passion fruit (*q*_max_ = 16 mg/g) for the adsorption of methylene blue dye from aqueous solutions [16]. HAp/chitosan composite with *q*_max_ = 769 mg/g is better than tamarind shell (*q*_max_ = 10.48 mg/g) and banana peels (*q*_max_ = 18.2 mg/g) for the adsorption of Congo red dye from aqueous solutions [16]. Anionic surfactant-modified activated carbon (ACMAS) with *q*_max_ = 235.7 mg/g [17] and sodium dodecyl sulphate-modified magnetic nanoparticles (SDS-MNPs) (*q*_max_ = 166.6 mg/g) [18] are better than avocado seed powder (*q*_max_ = 95.5 mg/g) and Haplophragma adenophyllum biomass (HAB) (*q*_max_ = 13.21 mg/g) [13] for the adsorption of GV dye from aqueous solutions. Holarrhena antidysenterica (HA) biowaste which is chemically treated with tartaric acid shows better adsorption for GV dye with *q*_max_ = 144.92 mg/g [14] than the nontreated (HA) biowaste (*q*_max_ = 128.2 mg/g) [14].

The main targets of this research are to investigate the potential of using unmodified HAp as an adsorbent for the removal of GV dye from aqueous solutions because there are no sufficient results in the literature about using it in the adsorption of GV dye from aqueous solutions and to estimate its effectiveness through comparison between its maximum adsorption capacity of GV dye and the other modified HAp adsorbents. Different experimental factors including contact time, adsorbent dose, initial concentration of GV dye, and pH were studied. In addition, surface characterization including SEM, EDX, and XRD of the prepared unmodified HAp adsorbent was performed in order to ensure the successful preparation using the combined precipitation microwave method. Also, FTIR surface characterization was performed before and after adsorption to identify the adsorption mechanism of GV dye using the unmodified HAp adsorbent.

## 2. Materials and Methods

### 2.1. Chemicals

All chemical reagents used in this study including calcium nitrate tetrahydrate (Ca(NO_3_)_2_.4H_2_O) with purity ≥99%, ammonium phosphate monobasic (NH_4_H_2_PO_4_) with purity ≥98.5%, ammonia solution (NH_4_OH, 30%), gentian violet (GV) dye (C_25_H_30_CIN_3_), sodium hydroxide (NaOH), and hydrochloric acid (HCl, 37%) were of analytical grade. These reagents were purchased from Sigma-Aldrich. Double-distilled water was used for the preparation of all solutions.

### 2.2. Synthesis and Characterization of Hydroxyapatite Adsorbent

Figure 1 represents the preparation scheme of the HAp adsorbent. Firstly, 0.02 M of calcium nitrate solution was prepared followed by stirring at room temperature and then 0.01 M of ammonium dihydrogen orthophosphate was added dropwise to this solution [19]. The pH of the mixture was measured as 5.44 and then it was adjusted to 9 by adding ammonium solution drop by drop followed by agitating the mixture using a magnetic stirrer for 24 h to allow the solution to precipitate [19]. The resulted precipitate was separated from the solution by centrifugation and washed many times using distilled water to get rid of all the nitrates and then it was dried using a microwave oven for 3 min [19]. Finally, the resulted material was grinded by a porcelain mortar to get the hydroxyapatite adsorbent as a powder [19].

The article "Kinetics and Isotherm Studies for Adsorption of Gentian Violet Dye from Aqueous Solutions Using Synthesized Hydroxyapatite" was published in 2023. Journal: J Environ Public Health.

### 2.3. Batch Experiments

Batch experiments were performed to determine the efficiency of the synthesized HAp adsorbent in the removal of the GV dye from aqueous solutions using four effecting factors including the pH of the solution, initial concentration, adsorbent dose, and contact time. The pH was studied in a range from 2 to 12 and the pH of samples were adjusted by using 0.1 M NaOH and 0.1 M HCl, the initial concentration of the GV dye was studied in a range of 1 mg/L–4 mg/L, the adsorbent dose was studied in a range of 0.2 g/L–2.5 g/L, and the contact time was studied in a range of 5 min–150 min. The removal efficiency of the GV dye was calculated by the following equation [20]:

(1) $$\begin{array}{c} removal\;efficiency\;\%=\left[\frac{\left(C_{o}\;–\;C\right)}{C_{o}}\right]*100\text{,} \end{array}$$

where *C*_o_ and *C* are initial and final concentrations of the GV dye in mg/L, respectively.

### 2.4. Equipment Used in the Preparation of HAp, Batch Adsorption Experiments, and Surface Characterization

During the preparation of the HAp adsorbent, a hotplate ceramic magnetic stirrer (Thermo-Fisher, USA) was used for stirring purposes with specifications of stirring ranging from 50 rpm to 1500 rpm and maximum surface temperature of 540°C. Also, a microwave model EM131MFF was used to dry the filtrate obtained from the agitation process after 24 h with specifications of power output of 1100 Watts and frequency of 2450 MHz. Batch adsorption experiments were performed in glass conical flasks that were shaken vigorously at 200 rpm using an orbital shaker model M49125 (Marshall Scientific, USA) with specifications of a speed interval from 24 rpm to 450 rpm. Upon shaking, the samples were separated using a centrifuge model D-37520 Osterode (Kendro Laboratory Products). The concentration of the GV dye in the filtered solutions was measured using a spectrophotometer (UV-5100, wavelength 190–1000 nm, Shanghai Metash Instruments, China). The morphology of the HAp adsorbent was determined by a scanning electron microscope (SEM) (Quattro S, Thermo Scientific, the Netherlands). X-ray diffraction (XRD) analysis for the HAp adsorbent was carried out using an Empyrean diffractometer (Malvern Panalytical, the Netherlands) with Ni-filtered Cu k*α* radiation (40 kV, 30 mA, and *λ* = 1.5406°A). The XRD analysis for samples was performed over a 2*θ* range of 4°–80°. The surface functional groups of HAp were recorded using Fourier transform infrared (FTIR) spectra (Vertex 70 RAM II, Germany).

The article "Kinetics and Isotherm Studies for Adsorption of Gentian Violet Dye from Aqueous Solutions Using Synthesized Hydroxyapatite" was published in 2023. Journal: J Environ Public Health.

### 2.5. Adsorption Kinetics Models

Adsorption kinetics models were used to determine the rate of adsorption which is used in the design of an adsorption system [21]. The experimental data of the GV dye adsorption on HAp were subjected to nonlinear forms of pseudo-first-order (PFO) and pseudo-second-order (PFO) models. Nonlinear regression using least square method was used for the calculation of kinetic parameters while using nonlinear equations. The nonlinear forms of the kinetic models PFO and PSO are described by the following equations [13, 14, 21]:

(2) $$\begin{array}{c} {PFO:q}_{t}=q_{e}*\left(1-e^{-K_{1}.t}\right)\text{,} \end{array}$$

(3) $$\begin{array}{c} {PSO:q}_{t}=\frac{K_{2}\;q_{e}^{2}\;t}{\left(1+K_{2}\;q_{e}\;t\right)}\text{,} \end{array}$$

where *q*_e_ and *q*_t_ (mg/g) are the amounts of the solute adsorbed by the adsorbent at equilibrium and at time (*t*), respectively. *k*_1_ (min^−1^) and *k*_2_ (mg/g.min) are rate constants for PFO and PSO, respectively.

During adsorption, the rate controlling step was observed by applying the intraparticle diffusion model. The intraparticle diffusion model is represented by the following equation [14, 15]:

(4) $$\begin{array}{c} q_{t}=k_{di\;ffusion}*t^{2}+C_{i}\text{,} \end{array}$$

where *q*_t_ (mg/g) is the amount of the solute adsorbed at time (*t*), *C*_i_ is the thickness of the layer, and *k*_diffusion_ is the adsorption rate constant of the intraparticle diffusion model.

### 2.6. Adsorption Isotherm Models

Adsorption isotherm models were used to determine the specific surface area, porosity, and maximum adsorption capacity for the solid adsorbent as these models describe the relation between the adsorbate in the liquid phase and the amount of adsorbate adsorbed on the solid surface of the adsorbent at equilibrium and at constant temperature [22]. The Langmuir, Halsey, and Dubinin–Radushkevich models were used to study the unmodified HAp adsorption system.

#### 2.6.1. Langmuir Isotherm

The Langmuir adsorption isotherm describes the equilibrium between the solid adsorbent and the adsorbate. This isotherm model is based on the assumption that the reactive groups are homogeneously distributed over the particulate's surface and that there is no lateral interaction. It is represented by the following equation [21, 23]:

(5) $$\begin{array}{c} q_{e}=\left(\frac{q_{m}*K_{L}*C_{e}}{1+\left(K_{L}*C_{e}\right)}\right)\text{,} \end{array}$$

where *C*_e_ and *q*_e_ represent the concentrations of the solute at equilibrium (mg/L) in solution and in solid phase (mg/g), respectively, *q*_m_ (mg/g) is the maximum monolayer adsorption capacity, and *K*_*L*_ (L/mg) is the Langmuir constant related to adsorption energy. *R*_L_ is the separation factor which gives an indication if the adsorption system is favorable to be fitted with the Langmuir isotherm model or not and it is calculated by the following equation [24]:

(6) $$\begin{array}{c} R_{L}=\frac{1}{1+K_{L}C_{o}}\text{,} \end{array}$$

where *C*_o_ is the initial adsorbate concentration (mg/g) [24]. *R*_L_ > 1 indicates unfavorable adsorption process, *R*_L_ = 0 indicates irreversible adsorption, *R*_L_ = 1 indicates linear adsorption, and 0 < *R*_L_ < 1 indicates favorable adsorption process [24].

The article "Kinetics and Isotherm Studies for Adsorption of Gentian Violet Dye from Aqueous Solutions Using Synthesized Hydroxyapatite" was published in 2023. Journal: J Environ Public Health.

#### 2.6.2. Halsey Isotherm

The Halsey isotherm is suitable for multilayer adsorption on a heterogeneous adsorbent surface [25]. The isotherm is represented through the following equation [25]:

(7) $$\begin{array}{c} qe=e^{\left(\ln K_{H}-\ln C_{e}\right)/n_{H}}\text{,} \end{array}$$

where *K_H_* and *n_H_* are the Halsey constants.

#### 2.6.3. Dubinin–Radushkevich Isotherm

The Dubinin–Radushkevich isotherm model is used to determine the porosity and apparent adsorption energy [26]. This model is mainly used to determine the mechanism of adsorption on heterogeneous surfaces: physical or ion exchange or chemical adsorption based on the value of the mean adsorption energy (*E*) [26]. This model is represented by the following equations [16, 27]:

(8) $$\begin{array}{c} q_{e}=q_{m}*e^{-\beta *{Ɛ}^{2}}\text{,} \end{array}$$

(9) $$\begin{array}{c} \epsilon =RT\;\ln\left(1+\frac{1}{C_{e}}\right)\text{,} \end{array}$$

(10) $$\begin{array}{c} E=\frac{1}{\sqrt{2\beta }}\text{,} \end{array}$$

where *ϵ* is the Polanyi potential, *β* (mol^2^/kJ^2^) is the Dubinin–Radushkevich constant, *R* is the gas constant (8.314 J/mol.k), *T* (K) is the temperature, and *E* (kJ/mol) is the mean adsorption energy.

### 2.7. Statistical Tests

To compare the application of different kinetics and isotherm models using nonlinear regression by the least squares method, the coefficient of determination (*R*^2^) and sum of square errors (SSE) were used as determining tools for the best-fit isotherm equations which can be calculated by the following equations [28]:

(11) $$\begin{array}{c} R^{2}=1-\frac{{\sum \left(q_{e,\exp}-q_{e,calc}\right)}^{2}}{{\sum \left(q_{e,\exp}-q_{e,mean}\right)}^{2}}\text{,} \end{array}$$

(12) $$\begin{array}{c} SSE=\overset{n}{\underset{i=1}{\sum }}{\left(q_{e,\exp}-q_{e,calc}\right)}^{2}\text{,} \end{array}$$

where *q*_e,exp_ (mg/g) is the experimental adsorption capacity at equilibrium, *q*_e,calc_ (mg/g) is the calculated adsorption capacity at equilibrium, and *q*_e,mean_ (mg/g) is the average of *q*_e,exp_.

The article "Kinetics and Isotherm Studies for Adsorption of Gentian Violet Dye from Aqueous Solutions Using Synthesized Hydroxyapatite" was published in 2023. Journal: J Environ Public Health.

### 2.8. Desorption and Regeneration of Cationic Dyes from HAp

Desorption experiments were essential in assessing whether the HAp adsorbent can be regenerated and reused in practical applications. For desorption experiments, several desorbing reagents have been reported for the desorption of cationic dyes such as methylene blue (MB) from various adsorbents, including acetic acid, HCl, KCl, and a mixture of methanol and acetic acid [29]. It has been reported that desorption of MB was achieved by placing poorly crystalline HAp in the phosphate solution after washing thoroughly with deionized water [29].

## 3. Results and Discussion

### 3.1. Characterization of Hydroxyapatite (HAp)

#### 3.1.1. Scanning Electron Microscopy (SEM) and Energy Dispersive X-Ray (EDX) Analyses

Figures 2(a) and 2(b) show the SEM images of the synthesized HAp adsorbent at two different scales 500 nm and 1 *μ*m, respectively, to show accurately its morphology where agglomerated spherical shape particles appeared on the surface. Also, the surface appeared quite irregular and porous.  Figure 3 shows the EDX analysis which ensured the presence of Ca, P, and O in the synthesized HAp crystallites. Atomic composition gave an acceptable Ca/P ratio of 1.43. The mentioned results were in agreement with the literature [30] ensuring the successful preparation of HAp.

#### 3.1.2. X-Ray Diffraction (XRD)

Figure 4 shows the XRD pattern of the synthesized HAp. It revealed that the substance was HAp crystallized in the hexagonal system with the parameters *a* = *b* = 9.4257 and *c* = 6.8853 Å which was in agreement with the literature [31] as the parameters of the hexagonal system of HAp were *a* = *b* = 9.41 Å and *c* = 6.931 Å proving the successful preparation of HAp adsorbent. Small peaks were appeared due to the presence of contaminants such as calcium hydroxide or calcium phosphates.

#### 3.1.3. Fourier Transform Infrared (FTIR)

Figure 5 shows the FTIR bands of HAp adsorbent before and after the adsorption of GV dye. On the basis of the FTIR bands of both cases, the positions of the vibration bands of 961.5 cm^−1^ and 1066.5 cm^−1^ were attributed to the phosphate of the HAp phase [32]. IR vibration bands at 742 cm^−1^ and 864 cm^−1^ were attributed to the carbonate functional group from the air [33]. The broad bands in the regions of 1639.3 cm^−1^ and 3351.8 cm^−1^ were attributed to the hydroxyl (OH^−^) group of adsorbed water molecules and the hydroxyl group, respectively [28].

The article "Kinetics and Isotherm Studies for Adsorption of Gentian Violet Dye from Aqueous Solutions Using Synthesized Hydroxyapatite" was published in 2023. Journal: J Environ Public Health.

As represented in Figure 5, shifting in peak positions of the PO_4_^3−^ group from 1066.5 cm^−1^ to 1074.2 cm^−1^, decrease in peak intensity of the PO_4_^3−^ group, disappearance of OH^−^ group peaks, and shifting in peak positions of the carbonate group from 742 cm^−1^ to 864 cm^−1^ were observed after the adsorption process ensuring that the adsorption of the GV dye was achieved successfully onto the HAp solid surface. This adsorption took place through the major functional groups of PO_4_^3−^, CO_3_^2−^, and OH^−^.

#### 3.1.4. Zeta Potential (ZP) Analysis

Zeta potential (ZP) is used to investigate the surface charging behavior of a solid material in contact with an electrolyte solution and it gives information about the point of zero charge (pH_pzc_) [34]. The main factor that affects the ZP is pH, and also there are other factors that affect the ZP including the ionic exchange, temperature, and viscosity of the medium [35]. ZP is indirectly measured through the following Henry's equation [34]:

(13) $$\begin{array}{c} \mu =\frac{2Єz}{3ղ0}\;f\left(ka\right)\text{,} \end{array}$$

where *μ* is the average electrophoretic mobility of the particle, *ε* is the relative permittivity of the medium, *z* is the average zeta potential, *η*_o_ is the dynamic viscosity of the medium, *k* is the reciprocal of the double layer thickness, and *a* is the radius of the spherical particle. The ratio of the particle radius to the electrical double layer thickness is given by the dimensionless parameter *ka*, which varies from 0 to ∞ [34]. The ZP potential is achieved as follows: when a material comes into contact with the electrolyte solution, a surface charge is developed at the interface. This phenomenon has different causes depending on the surface characteristics: in the case of hydrophobic surfaces with no functional groups, the exposed surface charge is due to the replacement of the adsorbed water molecules with ions (OH^−^ and H_3_O^+^); on the other hand, in the case of specific functional groups exposed on the surface, acid-base reactions between the liquid medium and these groups can take part (e.g., dissociation of the hydroxyl groups or protonation of the amine groups) with the consequent development of charges [35].

Figure 6 represents the point of zero charge (pH_pzc_) of the synthesized HAp adsorbent at a pH of 7.3 which was in agreement with the literature (around 7.9) [36]. As represented in Figure 6, the surface of the synthesized HAp was positively charged when pH was below the pH_pzc_ (7.3), so it could adsorb anionic dyes in this pH range. While the surface of the synthesized HAp was negatively charged when pH was above the pH_pzc_ (7.3), it could adsorb cationic dyes at this pH range. This ensured the ability of the synthesized HAp for adsorption in both acidic and basic mediums based on the nature of the adsorbate molecule.

The article "Kinetics and Isotherm Studies for Adsorption of Gentian Violet Dye from Aqueous Solutions Using Synthesized Hydroxyapatite" was published in 2023. Journal: J Environ Public Health.

### 3.2. Studying the Effect of Changing Parameters

#### 3.2.1. Effect of Contact Time

Adsorption experiments were performed at a contact time range of 5–150 min and under the following fixed conditions: pH = 12, initial dye concentration = 3 mg/L, and adsorbent dose = 1 g/L. As represented in Figure 7, the maximum dye removal percent (99.09%) was achieved at a contact time of 90 minutes, and beyond this time, the dye removal percent was almost unchanged. Therefore, the optimum contact time was considered to be 90 minutes.

#### 3.2.2. Effect of pH

Figure 8 shows that the maximum dye removal percentage reached its maximum value (99.32%) at pH = 12 and under the following fixed conditions: optimum contact time = 90 min, initial dye concentration = 3 mg/L, and adsorbent dose = 1 g/L. Therefore, the optimum pH was considered to be 12. As presented before, the surface of HAp was negatively charged when the solution's pH > pH_pzc_. Therefore, the GV dye adsorption on HAp was suggested to be described through the electrostatic interaction between the negatively charged surface of the HAp and the positively charged group of the dye. This electrostatic interaction mechanism in basic medium might be attributed to a strong hydrogen bonding via Lewis acid-base interaction between the (P-OH) and Ca^2+^ groups of the HAp adsorbent and the (N^+^) group found on the GV molecule as represented in Figure 9.

#### 3.2.3. Effect of Initial Dye Concentration

Figure 10 indicates that the GV dye removal percent increased from 80.25% to 99.32% with increase in initial dye concentration from 1 to 3 mg/L and under these fixed conditions: contact time = 90 min, pH = 12, and adsorbent dose = 1 g/L. The reason could be attributed to the chemical reaction occurrence between the adsorbent and the dye with increase in the initial dye concentration, but at the initial dye concentration of 3.5 mg/L, the dye removal percent decreased from 99.32% to 84.18% due to decrease in the active sites where the reaction between the adsorbent and the dye took place. As represented in Figure 10, the optimum initial concentration of GV dye was considered to be 3 mg/L at which the maximum dye removal percent (99.32%) was achieved.

Figure 11 represents a relation between the equilibrium adsorption capacity (*q*_e_) and the initial concertation of the GV dye (*C*_o_) where the equilibrium adsorption capacity increased from 0.8 mg/g to 2.99 mg/g for HAp with increase in the initial concentration of the GV dye from 1 mg/L to 3 mg/L. This could be attributed to an increase in the mass transfer driving force which accelerated the diffusion of GV ions from the bulk solution to the surface of HAp; this led to an increase in the equilibrium adsorption capacity and in the percent removal of the GV dye.

The article "Kinetics and Isotherm Studies for Adsorption of Gentian Violet Dye from Aqueous Solutions Using Synthesized Hydroxyapatite" was published in 2023. Journal: J Environ Public Health.

#### 3.2.4. Effect of Adsorbent Dose

Figure 12 represents that an increase in the adsorbent dose from 0.2 to 2.5 g/L had a positive effect on the GV dye removal percent as it increased from 92.78% to 99.1% under these fixed conditions: contact time = 90 min, pH = 12, and initial dye concentration = 3 mg/L. Excess increase in the adsorbent dose more than 1 g/L resulted in accumulation of HAp particles. Therefore, the specific surface area of the adsorbent decreased, and thus, the GV dye removal percent decreased from 99.1% to 73.32%. Therefore, the optimum adsorbent dose was considered to be 1 g/L at which the maximum dye removal percent (99.1%) was achieved.

### 3.3. Adsorption Kinetics

The adsorption kinetics of GV dye removal by HAp was studied at different levels of contact time ranging from 5 to 90 minutes and under the following fixed conditions: pH = 12, initial dye concentration = 3 mg/L, temperature = 25°C, and adsorbent dose = 1 g/L.

The results in Table 3 demonstrated that the PFO model was not suitable for the GV dye adsorption by HAp as the difference between the theoretical value of adsorption capacity at equilibrium (*q*_e,theoretical_) and the experimental value of adsorption capacity at equilibrium (*q*_e,experimental_) was higher than the difference in the PSO model. Also, the PSO model showed higher values for *R*^2^ and *K*_2_ (0.9996 and 0.730 mg g/min, respectively) than the PFO model (0.3679 and 0.563 min^−1^, respectively). In addition, the PSO model showed a lower value of SSE (0.0176) than the PFO model (0.0356). Therefore, GV dye adsorption from an aqueous solution by HAp was followed by the PSO model.

The rate controlling step for this adsorption system could be determined using the intraparticle diffusion model [37]. As represented in Figure 13, it was found that the plot of *q*_t_ vs. *t*^0.5^ gave almost a linear relation without division into two portions, indicating that the actual rate limiting step was the film diffusion.

### 3.4. Adsorption Isotherm

Adsorption isotherm models including the Langmuir, Halsey, and Dubinin–Radushkevich models were studied at different ranges of initial GV dye concentration from 1 mg/L to 3 mg/L and under the following fixed conditions: contact time = 90 min, pH = 12, and adsorbent dose = 1 g/L.  Table 4 shows that the Halsey isotherm model was best fitted with the experimental data compared with the Langmuir isotherm model because the value of SSE for the Halsey isotherm model (0.3489) was less than that for the Langmuir isotherm model (21.06). Also, the value of separation factor (*R*_L_) in the Langmuir isotherm model (1.19) was higher than 1 which indicated that the experimental data were unfavorable to be represented by this model. Therefore, the adsorption mechanism of GV dye using HAp was multilayer adsorption. The value of the mean adsorption energy (*E*) in the Dubinin–Radushkevich isotherm model was 8.45 kJ/mol, and this value was in between 8 kJ/mol and 16 kJ/mol which indicated that the adsorption process was achieved based on the electrostatic interaction between the surface of the adsorbent and the GV dye.

The article "Kinetics and Isotherm Studies for Adsorption of Gentian Violet Dye from Aqueous Solutions Using Synthesized Hydroxyapatite" was published in 2023. Journal: J Environ Public Health.

### 3.5. Thermodynamics Study

The nature of adsorption process whether it is spontaneous or nonspontaneous and the driving force of adsorption can be investigated through thermodynamics parameters of Gibbs free energy change (Δ*G*), enthalpy change (Δ*H*), and entropy change (Δ*S*) [3]. These parameters can be calculated from the following equations [3]:

(14) $$\begin{array}{c} ∆G=-RT\;lnk\text{,} \end{array}$$

(15) $$\begin{array}{c} k=\frac{C_{ad}}{C_{e}}\text{,} \end{array}$$

(16) $$\begin{array}{c} lnK=\frac{∆S}{R}-\frac{∆H}{RT}\text{,} \end{array}$$

(17) $$\begin{array}{c} ∆G=∆H-T∆S\text{,} \end{array}$$

where Δ*G* is the change in Gibbs free energy (kJ/mol.K), *R* is the universal gas constant (8.314 J/gmole.K), *T* is the temperature in Kelvin, *C*_ad_ is the concentration of solute in the solid adsorbent at equilibrium in mg/L, *C*_e_ is the concentration of solute in solution at equilibrium (mg/L), Δ*H* is the change in enthalpy (kJ/mol), and *k* is a thermodynamic constant [3]. Each of the following three different concentrations of GV dye of 1, 2, and 3 mg/L was studied at three different temperatures 20°C, 35°C, and 50°C under the following fixed conditions: pH = 12, adsorbent dose of 1 g/L, and contact time of 90 min, as represented in Table 5.

The values of Δ*H* and Δ*S* were determined by plotting “ln *k*” on the *y*-axis versus “1/*T*” on the *x*-axis to obtain the values of Δ*H* and Δ*S* from the slope and the intercept, respectively. Then, the values of Δ*G* were calculated from equation (17), as shown in Figure 14.

As represented in Table 6, it could be concluded that the adsorption process of the GV dye using the unmodified prepared HAp adsorbent was an endothermic process as the values of Δ*H* were positive. The negative values of Δ*G* indicated that this adsorption process was spontaneous. Also, it was noticed that at each initial dye concentration, the values of Δ*G* decreased with increase in temperature from 293 K to 323 K. This indicated that the process became more favorable at high temperatures.

The article "Kinetics and Isotherm Studies for Adsorption of Gentian Violet Dye from Aqueous Solutions Using Synthesized Hydroxyapatite" was published in 2023. Journal: J Environ Public Health.

## 4. Comparison of Adsorption Capacities of the Unmodified Prepared HAp Adsorbent with Other Adsorbents

The measuring key factor for the efficiency of an adsorbent in the uptake of any pollutant is its maximum adsorption capacity. The adsorption capacity of different adsorbents depends mainly on the source of the adsorbent, the process conditions of the adsorbent, and adsorbent modification. Due to the increasing demand of finding cheap adsorbents with high adsorption capacity, in the present study, a comparison was performed between the adsorption capacity of unmodified prepared HAp and other natural and modified adsorbents used in the adsorption of GV dye.  Table 7 presents the results of this comparison. The maximum adsorption capacity of rice husk ash (RHA) was 8.3 mg/g while the maximum adsorption capacity of charred rice husk (CRH) was 62.85 mg/g [38]. Also, the maximum adsorption capacities of activated carbon of lemon wood (ACL) and activated carbon of lemon wood (ACL)/Fe_3_O_4_ were 23.6 mg/g and 35.64 mg/g, respectively [36, 37]. As represented in Table 7, it could be concluded that the modification of adsorbents significantly increased their adsorption capacities. Also, Table 7 shows that the maximum adsorption capacities of hydroxyapatite (HAp) nanoparticles impregnated magnetic bentonite (HAp@Fe_3_O_4_@bentonite) composite and the unmodified HAp used in the present study were 1201.30 mg/g and 1.035 mg/g, respectively [40]. This indicated that the modified HAp has better adsorption capacity than the unmodified HAp.

## 5. Conclusions

The efficiency of the unmodified HAp for the adsorption of GV dye was found to be dependent on the contact time, initial dye concentration, pH, and adsorbent dose. Detailed surface characterization including SEM, EDX, and XRD was performed to ensure the successful preparation of HAp. In addition, FTIR surface characterization analysis was performed before and after the adsorption process and also the kinetics and isotherm models were studied to determine the adsorption mechanism. The PSO kinetic model was found to be the best model to describe the GV dye removal by HAp where the rate controlling step was the film diffusion. The Halsey isotherm model was the best fitted model with the experimental data to describe the GV dye adsorption system using HAp with a maximum adsorption capacity (*q*_max_) of 1.035 mg/g. The Dubinin–Radushkevich isotherm model indicated that the adsorption of GV dye from aqueous solutions was an adsorption process based on electrostatic interaction between the groups on the surface of the GV dye and the phosphate ions existing in an aqueous solution. Thermodynamic parameters were discussed to investigate the nature of the adsorption process of the GV dye from aqueous solutions at various temperatures and initial concentrations of GV dye. It was concluded that the adsorption process was endothermic due to the positive values of Δ*H* and spontaneous due to the negative values of Δ*G*. The optimum conditions for GV dye removal from aqueous solutions using the unmodified prepared HAp were investigated based on the performed batch adsorption experiments and the maximum dye removal percent (99.32%) was achieved at the following conditions: contact time = 90 min, pH = 12, initial dye concentration = 3 mg/L, and adsorbent dose = 1 g/L [41–44].

The article "Kinetics and Isotherm Studies for Adsorption of Gentian Violet Dye from Aqueous Solutions Using Synthesized Hydroxyapatite" was published in 2023. Journal: J Environ Public Health.

## 6. Future Research

Desorption batch experiments will be carried out in order to determine the number of cycles that the unmodified prepared HAp adsorbent can use. As part of the desorption experiments, various desorption reagents including phosphate solution, acetic acid, HCl, KCl, and methanol and acetic acid mixture will be applied to the unmodified HAp adsorbent to determine which reagent will be most effective to desorb the GV dye from the HAp adsorbent. In these batch experiments, kinetics and isotherms will be studied.

## Figures and Tables

**Figure 1:** Preparation scheme of the HAp adsorbent.

**Figure 2:** Scanning electron microscopy (SEM) of the synthesized HAp. (a) SEM image at a scale of 500 nm and (b) SEM image at a scale of 1 *μ*m. SEM analysis was used to illustrate the surface morphology.

**Figure 3:** EDX of the synthesized HAp. The EDX analysis shows the weight % for each element of the synthesized HAp.

**Figure 4:** XRD pattern of the synthesized HAp. The XRD analysis provides detailed information about the crystallographic structure, chemical composition, and physical properties of the synthesized HAp.

**Figure 5:** FTIR bands of HAp adsorbent before and after the adsorption of GV dye. FTIR analysis of the synthesized HAp is used to identify its chemical groups and changes occurred on them after the adsorption of phosphate ions from aqueous solutions.

**Figure 6:** Zeta potential analysis of the synthesized HAp adsorbent. Zeta potential analysis shows the surface charge of the synthesized HAp.

**Figure 7:** Effect of contact time on the GV dye removal percent. The GV dye removal percent increases with an increase in in the contact time.

**Figure 8:** Effect of pH on the GV dye removal percent. When pH > pH_pzc_, the GV dye removal percent increases while the GV dye removal percent decreases when pH < pH_pzc._

**Figure 9:** Schematic representation of the possible interactions between HAp and GV dye in the basic medium. This electrostatic interaction mechanism in basic medium may be attributed to a strong hydrogen bonding via Lewis acid-base interaction between the (P-OH) and Ca^2+^ groups of the HAp adsorbent and the (N^+^) group found on the GV molecule.

The article "Kinetics and Isotherm Studies for Adsorption of Gentian Violet Dye from Aqueous Solutions Using Synthesized Hydroxyapatite" was published in 2023. Journal: J Environ Public Health.

**Figure 10:** Effect of initial dye concentration on the GV dye removal percent. The GV dye removal percent increases with an increase in the initial concentration of GV dye, but to some extent at which more active sites are occupied with GV dye resulting in a decrease in the GV dye removal percent.

**Figure 11:** Relation between the equilibrium adsorption capacity (*q*_e_) and the initial concertation of GV dye. The equilibrium adsorption capacity (*q*_e_) increases with an increase in in the initial concentration of GV dye.

**Figure 12:** Effect of adsorbent dose on the GV dye removal percent. The GV dye removal percent increases with an increase in the adsorbent dose but to some extent at which agglomeration for adsorbents' particles occurred resulting in a decrease in the GV dye removal percent.

**Figure 13:** Intraparticle diffusion model for the adsorption of GV dye using HAp synthesized adsorbent. Intraparticle diffusion model shows the actual rate limiting step for the HAp-phosphate ion adsorption system.

**Figure 14:** Plot of (ln *k*) versus (1/*T*). From this plot, the values of Δ*H* and Δ*S* can be obtained from the slope and intercept, respectively.

**Table 1:** Maximum adsorption capacities of some agricultural wastes used for the removal of different dyes.

Adsorbents	Dye	*q*_max_ (mg/g)	References
Tamarind shell	Congo red	10.48	[12]
Banana peels	Congo red	18.2	[12]
Potato peels	Methylene blue	33.55	[12]
Avocado seed powder	Gentian violet	95.5	[12]
Yellow passion fruit	Methylene blue	16	[12]
Haplophragma adenophyllum biomass (HAB)	Gentian violet	13.21	[13]
Holarrhena antidysenterica (HA)	Gentian violet	128.2	[14]

**Table 2:** Maximum adsorption capacities of different adsorbents used for the removal of different dyes.

Adsorbents	Dye	*q*_max_ (mg/g)	References
HAp/chitosan composite	Congo red	769	[16]
HAp/hydrolyzed polyacrylamide 75	Methylene blue	435.6	[16]
Anionic surfactant-modified activated carbon (ACMAS)	Gentian violet	235.7	[17]
Sodium dodecyl sulphate-modified magnetic nanoparticles (SDS-MNPs)	Gentian violet	166.6	[18]
HA (tartaric acid treated)	Gentian violet	144.92	[14]

**Table 3:** Results of kinetics study.

Kinetic models	Parameters	Values
PFO	*q*_e_ (experimental) (mg/g)	2.973
	*q*_e_ (theoretical) (mg/g)	2.863
	*K*_1_ (min^−1^)	0.563
	*R* ^2^	0.3679
	SSE	0.0356

PSO	*q*_e_ (experimental) (mg/g)	2.973
	*q*_e_ (theoretical) (mg/g)	2.919
	*K*_2_ (mg/g. min)	0.73
	*R* ^2^	0.6876
	SSE	0.0176

The article "Kinetics and Isotherm Studies for Adsorption of Gentian Violet Dye from Aqueous Solutions Using Synthesized Hydroxyapatite" was published in 2023. Journal: J Environ Public Health.

**Table 4:** Results of adsorption isotherm.

Isotherm models	Parameters	Values
Langmuir	SSE	21.066
	*q*_max_ (mg/g)	0.722
	*K*_L_ (L/mg)	−0.054
	*R*_L_ (separation factor)	1.19

Halsey	SSE	0.3489
	nH	3.877
	*K*_H_ (L/mg)	0.434

Dubinin–Radushkevich	*β* (mol^2^/kJ^2^)	0.007
	*E* (kJ/mol)	8.45
	*q*_max_ (mg/g)	1.035

**Table 5:** Effect of changing temperature on the adsorption of GV dye.

Temperature (K)	Initial dye concentration (mg/L)	*C*_e_ (mg/L)	*C*_ad_ (mg/L)	*k*	ln *k*
293	1	0.11	0.89	8.09	2.09
	2	0.13	1.87	14.78	2.69
	3	0.0038	3	799	6.68

308	1	0.088	0.912	10.36	2.34
	2	0.092	1.908	20.71	3.03
	3	0.003	2.997	1194.22	7.09

323	1	0.075	0.925	12.33	2.51
	2	0.0912	1.9088	20.93	3.04
	3	0.0028	2.9972	1070.43	6.98

**Table 6:** Thermodynamics parameters for the adsorption of GV dye using the unmodified prepared HAp solid adsorbent.

Initial GV dye concentration (mg/L)	ln *k*	Temperature (K)	1/*T* (K*−*1)	Δ*H* (kJ/mol)	Δ*S* (kJ/mol.K)	Δ*G* (kJ/mol)
1	2.09	293	0.00341	11.08	0.06	−5.11
	2.34	308	0.00325			−5.94
	2.51	323	0.00310			−6.77

2	2.69	293	0.00341	9.26	0.05	−6.68
	3.03	308	0.00325			−7.50
	3.04	323	0.00310			−8.31

3	6.68	293	0.00341	7.88	0.08	−16.47
	7.09	308	0.00325			−17.72
	6.98	323	0.00310			−18.97

**Table 7:** Maximum adsorption capacities of different adsorbents used for GV dye removal.

Adsorbent	*q*_max_ (mg/g)	Ref
Charred rice husk (CRH)	62.85	[38]
Rice husk ash (RHA)	8.3	[38]
Activated carbon of lemon wood (ACL)	23.6	[38]
Activated carbon of lemon wood (ACL)/Fe_3_O_4_	35.64	[39]
Hydroxyapatite (HAp) nanoparticles impregnated magnetic bentonite (HAp@Fe_3_O_4_@bentonite)	1201.30	[40]
Unmodified hydroxyapatite (HAp)	1.035	This study

## Data Availability

The data used to support the findings of this study are available from the corresponding author upon request.
